# Clinical and Imaging Analysis of Cerebral Infarction Caused by Spontaneous Cerebral Artery Dissection Based on Augmented Reality Technology

This article has been retracted.

**DOI:** 10.1155/2021/6671121

**Published:** 2021-02-11

**Authors:** Yinghai Wang, Kedong Duan, Aihua Zhang, Yaping Lv, Dahai Cao

**Affiliations:** ^1^Internal Medicine Department, Dahua branch of Cangzhou Central Hospital, Cangzhou 061000, Hebei, China; ^2^Computer Tomography Room, Cangzhou Central Hospital, Cangzhou 061000, Hebei, China

## Abstract

In recent years, with the progress of population ageing, the incidence of a stroke caused by spontaneous dissection of the cerebral artery also increases with time. In order to address the health damage caused by a stroke caused by spontaneous dissection of the cerebral artery and to study its effect on human health, this article analyzes the incidence, type, electrocardiogram, and cardiovascular biomarker changes of cerebral infarction through statistical analysis and then discusses cerebral infarction. The pathogenesis and prevention measures of the disease are expected to provide better means for the treatment of cerebral infarction. Based on the case investigation of patients with cerebral infarction caused by spontaneous cerebral artery dissection, a case template was constructed, and a damage assessment matrix was created using a comprehensive quantitative and qualitative analysis method. Experimental results prove that cerebral infarction caused by spontaneous cerebral artery dissection is a great threat to human health, and the fatality rate of patients is extremely high. Enhanced imaging technology is of great help to clinical and image analysis, with a correlation coefficient of 0.87, compared with the other damage rate of cerebral infarction caused by spontaneous cerebral artery dissection which is about 15% higher than that of cerebral infarction caused by different methods. Studies have found that there are great differences in the age of people with cerebral infarction caused by spontaneous cerebral artery dissection, and the patients are generally over 45 years old. This shows that cerebral infarction caused by spontaneous cerebral artery dissection will cause great damage and affect people's health, which requires people's attention.

## 1. Introduction

Cerebrovascular disease is the first cause of death in my country and about 70% of cerebrovascular diseases are an ischemic stroke caused by acute brain artery obstruction. The incidence, mortality, and disability rate of the stroke are relatively high. The 75% of patients lost part of their workforce, bringing a great economic burden to the country and society [1]. The treatment of cerebral infarction emphasizes early detection, early diagnosis, early treatment, and early recovery to improve the prognosis and reduce the degree of disability of patients. The key to the treatment of cerebral infarction is vascular recanalization, which is obviously related to the improvement of clinical symptoms. With the development of augmented reality technology, it can improve the efficiency of vascular recanalization. The shorter the recanalization time, the better the clinical prognosis [2]. Patients with acute cerebral infarction should be admitted to the stroke unit for standardized treatment. A professional treatment team can greatly reduce the mortality and recurrence rate of patients with cerebral infarction.

Cerebral infarction is one of the more serious cerebrovascular diseases. Cerebral infarction has the characteristics of high incidence, high disability, and high fatality rate. This not only seriously endangers the public health and quality of life but also brings heavy social and economic burdens to the country and many families of patients [3]. Cerebral infarction is a common and frequently occurring disease that seriously endangers human health, with a high fatality rate and high disability rate, but there is no effective treatment method currently. Current research shows that the incidence of cerebral infarction ranks first in cerebrovascular diseases. Because the early prodromal symptoms of decreased blood supply to the brain tissue are not obvious, they usually manifest as dizziness and slight nausea, and these symptoms are often ignored by patients and eventually lead to cerebral infarction [4]. At present, many studies have shown that spontaneous cerebral artery dissection is related to the occurrence of cerebral infarction; that is, spontaneous cerebral artery dissection leads to a decrease in the blood supply of local brain tissue and then local brain tissue ischemic necrosis, and cerebral infarction occurs. Cerebral infarction is not entirely caused by spontaneous cerebral artery dissection. Studies have shown that the shedding of arterial plaque can also lead to the embolization of craniocerebral blood vessels and then cerebral infarction [5]. Experts at home and abroad have also conducted many studies on cerebral infarction caused by spontaneous cerebral artery dissection.

Liu Dongmei believes that spontaneous cerebral artery dissection is a very, very serious disease. It introduces the main manifestations and causes of spontaneous cerebral artery dissection and addresses the problems that spontaneous cerebral artery dissection is prone to occur in the diagnosis, such as misdiagnosis and missed diagnosis, and carried out related science popularization. After the patients were replaced with spontaneous cerebral artery dissection, they believed that treatment should be carried out in the early stage of symptoms to reduce the possible risk of patients [6] (Bian Yang). The clinical and image analysis of dissection analyzes the classification of patients with spontaneous cerebral artery dissection, classifies them according to gender, age, and so on and collects relevant information. It is believed that compared with cerebral infarction, the grade of patients with spontaneous cerebral artery dissection is lighter. Generally, there are no problems such as cerebral infarction and cerebral sclerosis. However, under the influence of external force, spontaneous cerebral artery dissection will be induced, which will cause the patient to change to cerebral artery dissection and cause the complications of cerebral infarction. For this situation, it is recommended that early diagnosis, early detection, early treatment, platelet aggregation, and anticoagulation therapy can be used to effectively prevent and treat [7]; Zhang Xiao chose to study acute cerebral infarction caused by cerebral artery dissection in the past 5 years. In the case of cerebral infarction, the characteristics of cerebral infarction caused by cerebral artery dissection were analyzed, and the infarct location and mechanism of the patient were analyzed. Zhang Xiao chose to study acute cerebral infarction caused by cerebral artery dissection in the past 5 years. In the case of cerebral infarction, the characteristics of cerebral infarction caused by cerebral artery dissection were analyzed, and the infarct location and mechanism of the patient were analyzed, and the relevant special diagnosis of the patient, such as gender, age, type of cerebral artery dissection, and dissection location, was done. A detailed record was made, and the pathogenesis and characteristics of cerebral artery dissection were analyzed, which provided a theoretical basis for the study [8]. These studies have a certain reference basis for this article. However, due to insufficient samples of these studies, too much emphasis on theories, and unreasonable practical schemes, the research has too many variables and the conclusions are unconvincing.

This article analyzes the advantages and disadvantages of previous studies and then proposes a model of cerebral infarction caused by spontaneous cerebral artery dissection based on augmented reality technology. This article mainly describes the basic characteristics and composition of the cerebral infarction caused by spontaneous dissection of the cerebral artery and the composition includes the use of a grid, the individual definition, the definition of status and action, and the interaction between individuals. Explain. The system objectively assessed the clinical relevance of spontaneous brain artery detection, explained the damage to the automatic dissection of the cerebral artery, and verified the preventive effect of enhanced reality technology on the spontaneous stroke that was caused by the dissection of the cerebral artery.

## 2. Cerebral Infarction Caused by Spontaneous Cerebral Artery Dissection Based on Augmented Reality Technology

### 2.1. Augmented Reality Technology

The continuous development of advanced reality technology has deepened the concept of virtual practice. Basically, the practice of enhanced reality technology continues to transform things into objective reality into digital image symbols through photoelectric and others and then express them in a virtual space. However, unlike the usual virtual practice, the practice in augmented reality makes the practice subject completely immersed in a virtual environment that can obtain real feelings, and through sophisticated sensing technology, people can obtain vision, hearing, touch, and smell that are the same as reality [9]. And the comprehensive feeling of kinesiology and then the motion tracker of various parts of the human body will feedback the subject's feedback into the virtual space. [10].

Augmented reality technology has brought about changes in human working life, entertainment and leisure, and practices. It has also brought about social issues such as excessive indulgence, health effects, violence, and value orientation and has spawned the evolution of the field of philosophy. The traditional philosophy of technology tends to study the various social effects of technology, but at the same time the development of technology will also have an impact on the philosophy system [11]. Affected by augmented reality technology, branches of philosophical fields such as artificial intelligence philosophy, virtual reality philosophy, and artificial life philosophy continue to appear. The philosophical issues generated by augmented reality technology involve many fields such as practical theory, media theory, epistemology, ethics, and sociology. Its unique technical characteristics and practical methods have produced different depths of utility in multiple disciplines [12].

The characteristics of augmented reality technology have caused philosophers to refocus on some traditional philosophical theories, such as the study of ontology and thinking about the nature of the world. Some brand-new philosophical ideas have emerged at the historic moment. In view of the technical characteristics of augmented reality that can construct a brand-new virtual environment, some scholars have put forward the idea that “computing” is the essence of the world. For example, the American philosopher Steinhart proposed digital metaphysics; Zhai Zhenming, a philosophy professor at Sun Yat-sen University in my country, proposed a new ethics, “world-making ethics,” and so on. Facing the continuous innovation of technology, philosophical thinking cannot stop but should lead and correct the new technology [13].

Since the advent of the Internet, virtual practice and augmented reality technology have attracted much attention. Through virtual practice and enhanced reality technology, humanity has transcended material production practice, social practice, and scientific practice, expanded the field of practice, increased knowledge objects, and improved practical ability. The development of augmented reality technology has added new vitality to virtual practice. If virtual practice is a practice that creates possibilities, then augmented reality practice is a practice that transforms any possibility into reality [14]. In the virtual environment, any condition becomes controllable. Human beings are no longer restricted by physiological, natural, and social factors and get rid of the shackles of material conditions. The digital symbol in the unit of bit abstracts the original concrete thing. In reality, the function of the thing is separated from the material carrier of the thing, and its function can be used alone anytime and anywhere without being restricted by the material carrier. This is no exception for humans. Augmented reality pulls human senses and consciousness out of the body, realizing truly beyond the limitations of time and space:

(1) $$\begin{array}{c} q=\beta *\partial *\left[{\left(\frac{t_{1}}{100}\right)}^{4}-{\left(\frac{t_{2}}{100}\right)}^{4}\right],\\ Q=\frac{\gamma }{t}A_{n}\left(T_{m}-T_{n}\right). \end{array}$$

For the application of augmented reality in the industrial field, Ian White, the responsible editor of the manufacturing section of the “Engineering” website, once said, “Factory planning, automation, assembly, maintenance, and training can all benefit from augmented reality [15].” With the continuous advancement of technology, augmented reality has become a practical tool for the manufacturing industry. Goldman Sachs Global Investment once predicted in a report that, by 2025, the revenue from augmented reality technology in the industrial sector will reach approximately US$4.7 billion. This is undoubtedly a contribution to augmented reality technology. The best value for industrial use is affirmed. Augmented reality can not only restrain the cost and integration of manufacturing [16] but also improve the effect of industrial design and the efficiency of training skills. Augmented reality is the most likely to bring forth one of the technologies of the subindustrial revolution; the industry 4.0 era has come to us [17].

### 2.2. Spontaneous Cerebral Artery Dissection

Cerebral artery dissection is a relatively rare disease in clinical practice [18]. The specific cause is currently unknown and the particular cause is currently unclear. Studies have confirmed that the inner rubber membrane and the middle rubber membrane of the brain artery dissection have suffered damage, but the specific pathological mechanism remains unclear. Cerebral arterial dissection is often missed due to the difficulty in recognizing imaging features. With the development of medical imaging technology, the diagnosis rate of cerebral arterial dissection has been improved, and there are more and more reports on cerebral arterial dissection. Cerebral artery dissection clinically mainly manifests as headache or symptoms related to cerebral infarction, subarachnoid hemorrhage, and compression symptoms. Studies have shown that patients with cerebral artery dissection can increase the incidence of clinical events through arterial-arterial embolism. And because the thrombus in the dissecting artery is a white thrombus with abundant platelets, anticoagulation and antiplatelet aggregation treatments are recommended clinically [6]. Anatomically, due to the lack of adequate supporting tissues such as the development of muscle fibers in the cerebral artery wall, the intracranial dissecting aneurysm is more common than the cerebral artery dissection, and it is more common in the vertebrobasilar system. Once the intracranial dissecting aneurysm is ruptured, it leads to subarachnoid hemorrhage, seriously endangers health, and is even directly threatening-life. Therefore, a high degree of vigilance is required clinically. Once a cerebral artery dissecting aneurysm ruptures, there is a high chance of rebleeding, so it usually requires surgery or interventional treatment:

(2) $$\begin{array}{c} \alpha =\frac{2.057f*{\left(v*p\right)}^{0.8}}{d^{0.2}},\\ T=\sqrt{\frac{{\left(a_{x1}-a_{x-1}\right)}^{2}+{\left(a_{y1}-a_{y-1}\right)}^{2}+{\left(a_{z1}-a_{z-1}\right)}^{2}}{100}}. \end{array}$$

There are corresponding imaging diagnostic guidelines for the early diagnosis of cerebral artery dissection, but there is no relevant guide or consensus on the best choice for the treatment of cerebral artery dissection. Clinicians generally treat the disease based on their own experience and expertise and select individualized treatment plan based on the specific condition of the patient. Intracranial artery dissections mostly occur in the vertebrobasilar artery, especially posterior circulation dissecting aneurysms, which are more prone to rupture and hemorrhage, which is extremely life-threatening. The treatment tends to be actively interventional or surgical treatment. Due to the difficulty of the posterior fossa surgical approach, active interventional therapy is the main treatment to stop bleeding quickly and prevent rebleeding [19].

### 2.3. Cerebral Infarction

Cerebral infarction, also known as ischemic stroke, is caused by limited cerebral ischemic necrosis or softening of brain tissue due to insufficient cerebral blood supply, hypoxia, and ischemia. The most widely used classification of cerebral infarction is TOAST classification, which is divided into 5 types: large artery atherosclerotic stroke, small artery occlusive stroke, cardiogenic cerebral embolism, and ischemic stroke caused by other reasons, Unexplained ischemic stroke, including large atherosclerotic stroke, namely, large atherosclerotic stenotic cerebral infarction, often leads to more serious consequences. Cerebral infarction is a short-term hypokinesia in the middle of the left ventricular wall caused by brain damage, with or without abnormal ventricular wall motion at the apex, and these abnormalities are completely restored in the subsequent course of the disease syndrome [20].

Cerebral infarction is mainly manifested by changes in electrocardiogram and abnormal cardiovascular biomarkers. The changes in ECG are the most common and obvious signs. It has been reported that 26%–73% of patients after cerebral infarction will have ECG changes, mainly including ischemic. Changes and arrhythmias, ischemic changes manifested as ST-T changes, acute myocardial infarction, pseudo myocardial infarction, and so on; arrhythmia manifested as QT interval prolongation, U wave, sinus tachycardia, sinus bradycardia, ventricular premature beats, atrial premature beats, paroxysmal atrial fibrillation, and so on, among which ischemic changes have the highest incidence; and one or several ECG abnormal changes can occur in the same patient [21].

Different parts of the brain injury can have different ECG changes because the brain has a direct regulatory effect on the heart. The insula has a representative area of the heart, and damage to the insula can affect visceral activities. In addition, the lateral and posterior regions of the hypothalamus can cause cardiac hyperresponsiveness. The medulla oblongata is the high-level center of breathing and heartbeat, and the central gray matter of the midbrain can directly regulate the heart. Damage can cause different types of arrhythmias [22].

The mechanism of cerebral infarction may be related to the central dysfunction of the hypothalamus, brainstem reticular structure, and limbic system (insula, etc.). In the acute phase of cerebral infarction, cerebral edema leads to increased intracranial pressure, which makes blood circulation disorders in the brain, hypothalamic edema, displacement, or ischemia and even affects the extensive and complex connection fibers between the hypothalamus and the thalamus, basal ganglia, and brainstem and causes autonomic nervous system dysfunction and impaired cardiac nerve mediation. In addition, in patients with acute cerebral infarction, the sympathetic nerve is excited. When the sympathetic nerve is excited, a large amount of catecholamines are released, which will accumulate in the myocardial tissue and cause secondary myocardial damage. This transmitter increases the excitability of cardiomyocytes and causes arrhythmia. Sinus tachycardia or supraventricular tachycardia can occur when acting on slow-reacting cells, and atrial (ventricular) arrhythmia can occur when acting on fast-reacting cells. Vascular endothelial cells increase the synthesis and secretion of endothelin and decrease the synthesis of nitric oxide, which further aggravates coronary artery spasm and myocardial ischemia [23]. At the same time, most patients with cerebrovascular disease have other risk factors, such as hypertension and diabetes. These factors play an important role in the occurrence and development of atherosclerosis. These patients may have coronary atherosclerosis and atherosclerosis before cerebral infarction. Myocardial ischemia induces or aggravates the abnormalities of ECG and cardiovascular biomarkers when the body is stressed [24].

### 2.4. Clinical Medicine

With the rapid development of digital medical care, electronic health data is increasing exponentially. How to make full use of the massive medical and health big data to improve the level and quality of medical and health services is one of the hot topics of current research. In order to ensure that early related functional exercises can be carried out after cerebral infarction caused by spontaneous cerebral artery dissection and reduce related postoperative complications, it is necessary to ensure the stability of the internal fixation, and the choice of treatment options for cerebral infarction caused by spontaneous cerebral artery dissection is not classified. In addition, consideration should also be given to age, damage, and other related comorbidities. For young patients, conservative treatment and surgical treatment can achieve better results. For elderly patients, it is recommended that conservative treatment requires a stage of debridement and drainage. After the wound is closed and there are no obvious signs of infection, second-stage surgical treatment is performed. With further analysis of the treatment of spontaneous cerebral artery dissection-induced cerebral infarction in the augmented reality technology, it is found that a good prognosis of spontaneous cerebral artery dissection-induced cerebral infarction is important for the follow-up rehabilitation which also plays an important role [25].

Due to poor blood supply to the brain, postoperative complications are mostly divided into early complications and long-term complications. The former mainly includes incision skin necrosis and incision infection, while the latter mainly includes abnormal healing and traumatic inflammation, which have serious impact. Therefore, in the surgical treatment of cerebral infarction caused by spontaneous cerebral artery dissection, it is necessary not only to make relevant preoperative preparations, to choose the correct surgical method and surgical approach, but also to reduce the surgical trauma under the premise of restoring reduction. The curative effect is improved and the patient's pain is relieved. After treatment, relevant prognostic treatment should be done to prevent various complications [26].

Augmented reality technology is the main development goal of technology realization and function realization [27]. In the current medical environment and actual rehabilitation treatment, how to understand and transform the expectations and needs of users more comprehensively, and how to integrate the form and structure of the product and function more in line with the needs of users are the focus of augmented reality technology. Its application in clinical medicine conforms to the following formula:

(3) $$\begin{array}{c} M=\frac{x}{\left(x+i+1\right)},\\ P_{LA}=L_{A}+\left[\frac{D_{A}-\left(L_{A}+1\right)}{C_{\text{skip}}\left(d\right)}\right]\times C_{\text{skip}}\left(d\right)+1,\\ d\left(x_{i},x_{j}\right)=\sqrt{\left({\left|x_{i1}-x_{j1}\right|}^{2}+{\left|x_{i2}-x_{j2}\right|}^{2}+...+{\left|x_{in}-x_{jn}\right|}^{2}\right)}. \end{array}$$

For the characteristics of the medical system, we have improved the relevant calculation functions:

(4) $$\begin{array}{c} f\left(i\right)=x_{0}+x_{1}y_{1}+x_{2}y_{2}+x_{3}y_{3},\\ W=\frac{N_{1}r_{1}^{2}}{2}+\frac{N_{2}r_{2}^{2}}{2}+N_{2}d_{2}^{2}+\left(\frac{N_{3}r_{3}^{2}}{2}+N_{3}d_{3}^{2}\right)*0.1+\frac{2}{3}N. \end{array}$$

## 3. Clinical and Imaging Experiments of Cerebral Infarction Caused by Spontaneous Cerebral Artery Dissection

### 3.1. Research Objects

Taking patients with cerebral infarction caused by spontaneous cerebral artery dissection in a city hospital as experimental subjects, collecting their clinical data (gender, age at diagnosis or diagnosis, clinical symptoms and signs at admission, auxiliary examinations including seven respiratory virus antigen tests, T lymphocytes subpopulation testing, allergen testing, fiberoptic bronchoscopy, BALF cytology count, lung function, lung CT, etc.), follow-up by telephone consultation and outpatient treatment. Performing retrospective analysis on the collected data and drawing conclusions are shown in Figure 1.

### 3.2. Experimental Purpose

Through the follow-up investigation of the patients, it is known whether the patient's condition is effectively controlled after the treatment of the cerebral infarction caused by spontaneous cerebral artery dissection and whether the control effect is obvious. We study the integrated medical system of the clinical disease and the brain block damage syndrome caused by spontaneous dissection of the cerebral artery and provide a report on the treatment of the immune system caused by a rheumatoid agent.

### 3.3. Statistics

All data analysis in this article adopts SPSS19.0 statistical test adopts two-sided test; significance is defined as 0.05, and *p* < 0.05 is considered as significant. The statistical results are displayed as mean ± standard deviation (*x* ± SD). When the test data complies with the normal distribution, the double T test is used for comparison within the group, and the independent sample T test is used for comparison between the groups. If the regular distribution is insufficient, two independent samples and two related samples will be used for inspection. The calculation formula is as follows:

(5) $$\begin{array}{c} d=\sqrt{\sum_{m=1}^{x}w_{n}*{\left(r_{nm}-uq_{m}\right)}^{2}},\\ d_{n}=\frac{1}{1+d\left(r_{n},uq\right)},\\ P=\sqrt{\frac{\sum_{a=1}^{a=x}{\left(Rf\left(W\left(\gamma_{a}\right)\right)-Rf\left(W_{0}\left(\gamma_{a}\right)\right)\right)}^{2}}{\sum_{a=1}^{a=x}{\left(RfW_{0}\left(\gamma_{a}\right)\right)}^{2}}.} \end{array}$$

## 4. Clinical and Imaging Analysis of Cerebral Infarction Caused by Spontaneous Cerebral Artery Dissection

### 4.1. Distribution of Patients

We collected statistics on people who had undergone treatment for cerebral infarction caused by spontaneous cerebral artery dissection in city hospitals and classified them according to factors such as age and gender. We hope to find out the characteristics and regularities of cerebral infarction caused by spontaneous cerebral artery dissection. The specific patient data are shown in Table 1.

According to Figure 2 and Figure 3, we can see that the probability of cerebral infarction caused by spontaneous cerebral artery dissection is different between different ages. The population of cerebral infarction caused by spontaneous cerebral artery dissection is mainly distributed in the young and middle-aged, namely, 45 years old. In the following, of a total of about 540 people, accounting for more than the general population of this survey, and for people over 60 years old, the number of radius fractures is about 150, accounting for about 17% of the total number. This indicates that cerebral infarction caused by spontaneous cerebral artery dissection mainly occurs in young and middle-aged people, and related treatment methods should also be tilted towards the side. We have investigated patients with other causes of cerebral infarction, as shown in Table 2.

From Figure 4, we can see that, unlike spontaneous cerebral artery dissection caused by cerebral infarction, the age of cerebral infarction in general patients is too old, and more than 70% of them are over 45 years old, while spontaneous cerebral artery dissection causes cerebral infarction. The age distribution is relatively uniform, and there are many young and middle-aged patients. This is because the triggers of cerebral infarction caused by spontaneous cerebral artery dissection are different from other cerebral infarctions. Cerebral infarction caused by spontaneous cerebral artery dissection is generally caused by external factors, so the age change is not obvious.

### 4.2. Treatment Methods

For cerebral infarction caused by spontaneous cerebral artery dissection, the current treatment methods include drug treatment, anticoagulation treatment, platelet aggregation treatment, vascular medical treatment, and the method of augmented reality technology used in this article. We make statistics on the current treatment population; the detailed data is shown in Table 3.

From Figure 5, we can see that, for the vast majority of patients, using augmented reality technology in conjunction with other treatment methods is not the first choice. This is because this method requires more steps and is less severe to cerebral infarction. People who are more inclined to choose medication or other treatment methods. However, with the development of time, augmented reality technology and treatment have been more and more accepted by people. We have collected data from 2010 to 2019, as shown in Table 4.

It can be seen from Figure 6 that over time, the treatment of cerebral infarction has also undergone certain changes. Although conservative treatment is still the first choice for the treatment of cerebral infarction according to patients, in recent years, the use of augmented reality technology to cooperate with treatment has been recognized and tried by more and more people, and the increase rate is about 18%, which is gradually accepted by people.

### 4.3. Effects of Different Treatment Methods

For cerebral infarction caused by spontaneous cerebral artery dissection, the treatment effect is the most concerned issue for patients. We have carried out quantitative calculations on different treatment methods through the calculation models mentioned in the article and carried out relevant statistics. According to the calculation results, the final value is above 0.8 for excellent healing effect, and the value above 0.5 is passed. The specific statistical results are shown in Table 5.

It can be seen from Figure 7 that the scores of the methods in this article are basically higher than those of other methods, and the stability and pain-free sensation are both above 0.8 points. Compared with other methods, the combined treatment with augmented reality technology can not only remain stable during treatment, but also perform extremely well in other areas. The prognostic treatment of cerebral infarction caused by spontaneous cerebral artery dissection is also extremely important. For this, we have counted several important prognostic indicators, which are shown in Figure 8.

We can see from Figure 8 that, in terms of prognosis, the use of spontaneous cerebral artery dissection to treat cerebral infarction combined with treatment of cerebral infarction also has many advantages in prognostic treatment, and its score is basically maintained above good. Although other methods have their own advantages, in general, the cooperation of spontaneous cerebral artery dissection-induced cerebral infarction can play an important role in the treatment and prognosis.

## 5. Conclusions

This study mainly focused on changes in cardiovascular biomarkers. In the selection of inclusion criteria, we tried to exclude other factors that can affect heart function and patients with previous heart diseases. However, patients with cerebrovascular diseases mostly have various heart and brain diseases. Vascular risk factors may interfere with the results of the study. In addition, in the study of the influence of the infarct position on the ECG and cardiovascular biomarkers, due to the small sample size of this study and the large number of groups, the reliability of the research results needs to be verified by a larger sample size.

Patients can improve or control the increase in blood pressure and low-density lipoprotein through exercise or changing their diet and reduce smoking or quit smoking, which can effectively prevent the occurrence of cerebral infarction. In addition, high blood pressure and low-density lipoprotein can also be used as predictors of cerebral infarction to detect the blood pressure and low-density lipoprotein indicators of patients with spontaneous cerebral artery dissection. If abnormalities are found and can be well controlled and improved, it may prevent the brain occurrence of infarction. For clinical work, doctors can more simply and intuitively guide patients to prevent cerebral infarction after carotid artery stenosis, which is of great help in preventing cerebral infarction caused by spontaneous cerebral artery dissection.

In future studies on cerebral infarction caused by spontaneous cerebral artery dissection, more assessment indicators of autonomic nerve function should be collected, such as heart rate variability and changes in catecholamine concentration; in addition, evaluation of the central autonomic nervous system should also be included. It requires the joint efforts of neurology, cardiology, neuroimaging, neurophysiology, and other disciplines to promote research in this field, with a view to formulating standardized treatment methods for postcerebral infarction prevention and control, which will improve cerebral infarction. The clinical prognosis of patients is very important to reduce mortality.

## Figures and Tables

**Figure 1:** Experimental inspection items.

**Figure 2:** Population distribution.

**Figure 3:** Age distribution of radius fractures.

**Figure 4:** Age distribution of radius fractures.

**Figure 5:** Radius fracture treatment.

**Figure 6:** The difference in treatment in different years.

**Figure 7:** Treatment effect of different methods.

**Figure 8:** Prognostic treatment score.

**Table 1:** Cerebral infarction caused by spontaneous cerebral artery dissection.

Age	Minor cerebral infarction	General cerebral infarction	Severe cerebral infarction	Very severe cerebral infarction	Extremely serious infarction
0–12	3	8	11	7	8
13–26	66	88	31	47	18
27–45	57	61	99	36	26
46–60	32	91	87	53	13
Over60	27	42	51	21	9

**Table 2:** Other causes of cerebral infarction.

Age	Minor cerebral infarction	Cerebral infarction	Severe cerebral infarction	Very severe cerebral infarction	Extremely serious infarction
0–12	1	1	2	4	1
13–26	17	22	26	15	14
27–45	42	35	47	39	33
46–60	47	52	49	53	59
Over 60	63	67	72	61	54

**Table 3:** Difference in treatment.

	Thrombolytic therapy	Anticoagulant therapy	Platelet aggregation therapy	Vascular medicine treatment	Augmented reality technology
Minor cerebral infarction	3	29	47	31	21
Cerebral infarction	1	21	51	26	13
Severe cerebral infarction	26	54	63	47	19
Very severe cerebral infarction	5	19	27	29	15
Extremely serious infarction	2	36	19	26	12

**Table 4:** Difference in treatment.

	2010	2011	2012	2013	2014	2015	2016	2017	2018	2019
Thrombolytic therapy	37	44	49	66	57	63	75	51	47	42
Anticoagulant therapy	19	21	27	33	51	47	41	39	46	41
Platelet aggregation therapy	67	72	79	69	88	109	97	89	81	76
Vascular medicine treatment	29	36	33	42	39	33	45	47	56	55
Augmented reality technology	1	3	9	15	13	17	23	26	33	37

**Table 5:** Treatment effect of radius fracture.

	Stability	Thalamus	Brain stem	Pain	Cerebellum	Recovery effect
Thrombolytic therapy	0.537	0.887	0.528	0.71.8	0.642	0.516
Anticoagulant therapy	0.431	0.573	0.431	0.752	0.669	0.678
Platelet aggregation therapy	0.479	0.526	0.888	0.697	0.477	0.617
Vascular medicine treatment	0.539	0.643	0.542	0.573	0.681	0.854
Augmented reality technology	0.879	0.735	0.779	0.727	0.813	0.795

## Data Availability

No data were used to support this study.

## References

[1] Liu D., Xin X., Zhang J. (2020). A case of cerebral infarction-aortic dissection-related cerebral infarction caused by complex etiology. *Frontiers of Medicine*.

[2] Li F., Zhang S. (2018). One case report of cerebral infarction caused by unilateral internal carotid artery dissection. *Medical Information*.

[3] Wang C., He Z., Huang J. (2016). A case of cerebral infarction caused by internal carotid artery dissection after exercise. *Guangdong Medical Journal*.

[4] Wang L., Jin K., Wu J. (2016). A case of acute cerebral infarction caused by spontaneous recanalization of atherosclerotic internal carotid artery occlusion. *Chinese Journal of Emergency Medicine*.

[5] Chen H., Li Z., Hong H. (2016). Analysis of clinical and imaging characteristics of 118 cases of spontaneous cerebral artery dissection caused by ischemic stroke. *Chinese Journal of Internal Medicine*.

[6] Yu S., Zhou J. (2020). Efficacy analysis of emergency endovascular stenting for acute cerebral infarction caused by carotid artery dissection. *Stroke and Nervous Diseases*.

[7] Zhao K., Wang J., Fang Y. (2018). The prognosis and influencing factors of unruptured intracranial spontaneous vertebral artery dissecting aneurysm with stent reconstruction technique. *Chinese Journal of Neurosurgery*.

[8] Ye F., Wang Z., Pan X. (2017). Spontaneous bilateral internal carotid artery dissection: a case report and literature review. *Chinese Journal of General Practitioners*.

[9] Lv Z., Halawani A., Feng S., Réhman S., Li H. (2015). Touch-less interactive augmented reality game on vision-based wearable device. *Personal and Ubiquitous Computing*.

[10] Wu J. (2019). A case of intravenous thrombolytic therapy for cerebral infarction caused by spontaneous carotid artery dissection on the left side. *China Rural Medicine*.

[11] Xiang Z., Cao W., Zhang H. (2017). Diagnosis and treatment of cerebral infarction caused by bilateral internal carotid artery dissection. *Journal of International Neurology and Neurosurgery*.

[12] Liang W., Ou Z., Zhang W. (2017). A successful mechanical thrombectomy for cerebral infarction caused by internal carotid artery dissection and internal carotid artery/middle cerebral artery occlusion after awakening and literature review. *Practical Journal of Cardio-Cerebral Pneumal and Vascular Disease*.

[13] Xiao C., Chen B. (2019). Analysis of the use of antithrombotic drugs in a case of intracranial hemorrhage secondary to cerebral infarction caused by acute internal carotid artery dissection. *Pharmacy Today*.

[14] Hu Y., Zhao C. (2020). A case of forensic identification of cerebral infarction caused by traumatic carotid artery dissection. *Chinese Journal of Forensic Medicine*.

[15] Tang L., Yu Z., Zhang D. (2016). Analysis of risk factors and etiology of young cerebral infarction. *Laboratory Medicine and Clinics*.

[16] Tsai S.-B., Lee Y.-C., Wu C.-H., Guo J.-J. (2013). Examining how manufacturing corporations win orders. *South African Journal of Industrial Engineering*.

[17] Zhu Y., Ding X., Ying W. (2016). Combined diagnosis of internal carotid artery dissection by carotid artery ultrasound and transcranial color Doppler. *Prevention and Treatment of Cardiovascular and Cerebrovascular Diseases*.

[18] Shankar K., Elhoseny M., Lakshmanaprabu S. K. (2020). Optimal feature level fusion based ANFIS classifier for brain MRI image classification. *Concurrency and Computation: Practice and Experience*.

[19] Fang Y., Chang J., Niu X. (2017). Clinical characteristics, treatment and follow-up of 42 cases of carotid artery dissection. *Journal of Shanxi Medical University*.

[20] Yan J., Yan X., Wang Y. (2017). A case report of thoracic-abdominal aortic dissection resembling acute cerebral infarction. *Journal of Apoplexy and Nervous Diseases*.

[21] Liu D., Zou H., Hao Y. (2018). A case report of aortic dissection with cerebral infarction onset. *Apoplexy and Nervous Diseases*.

[22] Tan X., Du D., Tan (2017). Clinical characteristics of arterial dissection and large atherosclerotic cerebral infarction and analysis of cerebrovascular angiography results. *Laboratory Medicine and Clinics*.

[23] Shen L., Xie F., Du T. (2016). Ultrasound diagnosis of ascending aorta, brachiocephalic trunk, and right common carotid artery dissection with cerebral infarction in 1 case. *Journal of Clinical Ultrasound in Medicine*.

[24] Liu S., Cao X., Zhao J. (2017). Recanalization of anti-platelet aggregation therapy in extracranial internal carotid artery dissection and review of literature. *Jiangxi Medicine*.

[25] Qiao L., Liu X. (2016). Two cases of acute aortic dissection with cerebral infarction as the primary manifestation. *People’s Army Surgeon*.

[26] Yu H., Feng K. (2018). Analysis of clinical characteristics of acute aortic dissection combined with acute cerebral infarction. *Chinese Journal of Geriatric Cardiovascular and Cerebrovascular Disease*.

[27] Zhang W., Ning B., Li X. (2019). High-resolution magnetic resonance imaging of intracranial arteries in patients with acute cerebral infarction. *Journal of Apoplexy and Nervous Diseases*.

